# Occupational Health Development and Safety Management of Enterprise Employees Based on the Perspective of Sustainable Environment

**DOI:** 10.1155/2022/3792356

**Published:** 2022-09-08

**Authors:** Qilong Chen, Hongliang Li, Xiao Pan

**Affiliations:** ^1^College of Marxism, Nanjing University of Science and Technology, Nanjing 210000, Jiangsu, China; ^2^Glorious Sun School of Business and Management, Donghua University, Shanghai 200000, China; ^3^School of Business, Nantong Institute of Technology, Nantong 226000, Jiangsu, China

## Abstract

In recent years, the economy of enterprises has developed rapidly. Most enterprises focus on economic interests and ignore the occupational health of employees, resulting in an increase in the occupational morbidity rate of employees. Occupational insecurity of corporate employees will reduce the work efficiency of employees. In turn, it will affect the economic development of the enterprise. Paying attention to the occupational health and safety development of corporate employees is a necessary measure for corporate economic development. The main reasons that endanger the occupational health of employees are the unreasonable discharge of pollutants and the substandard treatment of pollutants. The sustainable environmental strategy of enterprise development can well control the risk factors that endanger the occupation of enterprise employees, and it is conducive to the health and safety development of enterprise employees and enterprises. This paper studied the impact of sustainable environmental factors on the occupational health and safety development of enterprise employees through the fuzzy analytic hierarchy process and analyzed the impact on the occupation of enterprise employees according to the larger influencing factors. The experimental results showed that heavy metal wastewater, dust, hydrogen sulfide gas, and high-temperature radiation are the four most weighted impact indicators. Different concentrations of these four indicators are tested; when the concentration value of these impact indicators is low, it has little impact on the occupational safety and development of enterprise employees. However, when the concentration increases, the occupational safety and development of enterprise employees are seriously reduced. When the safety is the lowest, it is only 20%, and the development is only 23%. Carrying out sustainable environmental development can reduce the discharge of industrial waste; hence, while protecting the environment, the occupational health and safety and development potential of employees can be improved.

## 1. Introduction

Under the influence of the Industrial Revolution, human production and life have developed rapidly, and industrialized industries have brought people a lot of convenience. Early enterprises did not pay attention to the protection of the environment in the production process, which led to the random discharge of pollutants from the enterprise. And the employees of the enterprise would inevitably inhale the pollutants discharged by the enterprise, causing serious bodily harm to them. In recent decades, the excessive exploitation of natural resources by enterprises has forced the employees of enterprises to overwork, which has seriously affected the occupational safety of employees. Even in some enterprises, the excessive mining of radioactive elements has damaged the environment and caused irreparable harm to employees. There are serious problems in the occupation of enterprise employees. Only by following the sustainable development strategy can the enterprise develop the occupational health and safety of enterprise employees. By analyzing which factors from the perspective of sustainable environment have an impact on the occupational health and safety management of employees, different measures can be implemented according to different situations of the enterprise to ensure the occupational health and safety development of enterprise employees. Therefore, this paper has research significance.

There are many dangerous problems in the occupation of enterprise employees. The relevant researchers have analyzed the occupational health development and safety management of enterprise employees. Among them, Evangelinos et al. analyzed the occupational safety issues of employees in 50 large enterprises. The employee injury rate of enterprises that implement the occupational health development and safety management strategy of enterprise employees will be relatively lower, which is conducive to the career development of the company's employees [1]. Almost et al. found that by establishing a safety management system for the occupational health and development of employees, the company's annual investment in employee injuries was greatly reduced [2]. Fagbe et al. pointed out that the occupational health development and safety management of enterprise employees can reduce the risk of employee injury and improve the economic benefits of enterprises [3]. Mouras and Badri showed that, in some industrial enterprises, occupational health development and safety management is very necessary, which can effectively protect the safety of enterprise employees [4]. Skad used the method of fuzzy analysis to improve the effectiveness of occupational health development and safety management of enterprise employees [5]. The application of occupational health development and safety management can effectively reduce the probability of employee injury and improve employee occupational safety, but there is a lack of in-depth research on specific directions.

The natural environment affects the occupational safety development of enterprise employees, and the occupational health development and safety management of enterprise employees in a sustainable environment is studied. Among them, Marzaleh et al. pointed out that the development of sustainable environment can improve the occupational safety of enterprise employees [6]. Research of Mohammadfam et al. showed that there is a coupling relationship between the environment and the occupation of enterprise employees, and the occupational healthy development of enterprise employees must rely on a sustainable environment [7]. A sustainable environment can effectively improve the efficiency of the occupational health development of enterprise employees. Jilcha and Kitaw believed that sustainable development to improve environmental issues can help employees to bring more development potential [8]. Sarkheil pointed out that a sustainable environment can provide better safety and development for the career of enterprise employees [9]. Shammi et al. believed that by reducing the discharge of industrial waste liquid and adhering to the principle of sustainable environment, the occupational health and safety development of employees can be improved [10]. Although a sustainable environment can improve the occupational health and safety development of employees, there is a lack of evaluation methods to qualitatively or quantitatively analyze the occupational health and safety management of employees in a sustainable environment.

Sustainable environmental development and occupational health and safety management of employees are related to each other. The factors that affect the occupational health and safety development of enterprise employees are analyzed. Corresponding measures are taken to improve the efficiency of occupational health and safety development of employees in the enterprise according to the relevant factors analyzed [11]. The innovation point of this paper is as follows: using fuzzy analytic hierarchy process to analyze the related factors of sustainable environment and occupational health development and safety management of enterprise employees.

## 2. Methods of Relevance Evaluation of Occupational Health Development

In the current enterprise form, enterprises should not only focus on improving the economic benefits of the enterprise but also pay more attention to the employees of the enterprise. The competition between enterprises is actually the competition among the employees of the enterprise and the competition of the positions of the enterprise. In the process of development, the enterprise can effectively improve the comprehensive ability of the enterprise by carrying out the healthy development and safety management of the occupation of the enterprise employees [12]. The sustainable environmental policy is a strategy to effectively reduce the pollutant discharge of the enterprise. It can effectively affect the occupational health development and safety management of employees [13]. The evaluation and analysis of indicators for the occupational health development and safety management of enterprise employees from the perspective of sustainable environment can effectively improve the occupational safety of enterprise employees. From the perspective of sustainable environment, the occupational health development and safety management structure of enterprise employees is shown in Figure 1.

It can be seen from Figure 1 that the sustainable environment and the occupational health development and safety management of employees of the enterprise work together and develop together. Therefore, it is very important to analyze the occupational health development and safety management of enterprise employees from the perspective of sustainable environment. Common evaluation and analysis methods include AHP, percentile analysis, fuzzy analysis, and fuzzy AHP [14].

### 2.1. Analytic Hierarchy Process

Analytic hierarchy process (AHP) is a qualitative and quantitative analysis method for complex model problems, which can be well applied to the occupational health development and safety management of enterprise employees from the perspective of sustainable environment [15]. It mainly decomposes complex problems, compares the decomposed indicators with mathematical methods, determines the weight of the indicators, and then realizes the quantitative analysis of multiple indicators of the research system. The structural model of AHP is shown in Figure 2.

The general steps of AHP are as follows: decomposing the analysis system according to the level, testing the validity of each level and the overall analysis data, and analyzing the weight of each index. The first layer of the analytic hierarchy process is the goal to be achieved by the system. In this paper, it is the occupational health development and safety management of enterprise employees. The second layer is the preliminary analysis of the goal, and the third layer is the specific analysis of the goal. There is a subordinate relationship between layers, and the indicators between layers are independent of each other [16].

The analysis of AHP usually requires the help of judgment matrix. The judgment matrix is a method for weight analysis of each index in the index layer, and it is a way of quantitative analysis. The process of using the judgment matrix in AHP is as follows:

Let there be *n* indicators *S*={*s*_1_, *s*_2_,…, *s*_*n*_}, taking the influence of any two indicators *s*_*i*_ and *s*_*j*_ on the target, and using element *k*_*ij*_ in the matrix to represent the ratio between the two indicators. Therefore, the judgment matrix can be expressed as follows:

(1) $$\begin{array}{c} K={\left(k_{ij}\right)}_{n\times n}. \end{array}$$

Here, *k*_*ij*_ represents the influence ratio of the *i*th indicator and the *j*th indicator.

Then, in turn, the ratio of the influence of the *j*th indicator to the *i*th indicator is as follows:

(2) $$\begin{array}{c} k_{ji}=\frac{1}{k_{ij}}. \end{array}$$

The setting of the median value of the judgment matrix is the analysis basis of the judgment matrix. And the setting rule of the median value of the judgment matrix is a scoring rule. The meaning of the judgment matrix is shown in Table 1.

The process of validating the judgment matrix is as follows:

The maximum eigenvalue of the judgment matrix needs to be solved, and the solving process is a matrix solving method. The maximum eigenvalue is set to *μ*_max_.

Then, the index of validity test can be expressed as follows:

(3) $$\begin{array}{c} A=\frac{\mu_{\max}-n}{n-1}. \end{array}$$

Here, *n* represents the total number of indicators.

Find the corresponding effectiveness index:

(4) $$\begin{array}{c} B=\frac{\mu_{\max}^{\prime }-n}{n-1}. \end{array}$$

Here, *μ*_max_′ is the average maximum eigenvalue of the judgment matrix.

Then, the validity ratio of the judgment matrix can be expressed as follows:

(5) $$\begin{array}{c} R=\frac{A}{B}. \end{array}$$

When *R* is less than 0.1, the judgment matrix is considered to be valid; on the contrary, the judgment matrix is invalid.

The calculation of the weight of each index adopts the arithmetic mean solution method, that is, the arithmetic mean of each column vector in the judgment matrix represents the weight of the index. The formula is expressed as follows:

(6) $$\begin{array}{c} v_{i}=\frac{k_{i1}+k_{i2}+\cdots +k_{in}}{n}. \end{array}$$

Here, *v*_*i*_ represents the weight of the *i*th index.

AHP is widely used in analyzing, evaluating, and predicting the target system under study due to its advantages of simple design and quantitative analysis.

### 2.2. Percentile Analysis

It is a scoring mode based on the initial value of the index and the weight of the index, and the impact on the occupational health development and safety management of the employees of the enterprise is reflected through the score. The higher the score, the greater the impact of this indicator on the occupational health development and safety management of employees. The evaluation process of the percentile analysis method is as follows:

Let the decision-making set be *B*={*b*_1_, *b*_2_,…, *b*_*m*_}, the indicator set be *C*={*c*_1_, *c*_2_,…, *c*_*m*_}, the judge set be *R*={*r*_1_, *r*_2_,…, *r*_*h*_}, and the score of the judge *i* to the index *j* be *s*_*ij*_.

Then, the average score for indicator *j* is as follows:

(7) $$\begin{array}{c} {\bar{s}}_{j}=\frac{1}{h}\sum_{i=1}^{h}s_{ij}. \end{array}$$

Here, *h* represents the total number of judges.

The scoring deviation for metric *j* is as follows:

(8) $$\begin{array}{c} e_{ij}=\left|s_{ij}-{\bar{s}}_{j}\right|. \end{array}$$

Here, the smaller the value of *e*, the more accurate the evaluation.

Standardize on scoring bias:

(9) $$\begin{array}{c} g\left(e_{ij}\right)=\frac{e_{ij}-\min e_{ij}}{\max e_{ij}-\min e_{ij}}. \end{array}$$

Then, the objective score of the judge can be expressed as follows:

(10) $$\begin{array}{c} M=\sum_{i=1}^{m}g\left(e_{ij}\right). \end{array}$$

Let the judge's fairness be *N*.

Then, the criteria of the judges for the indicators are as follows:

(11) $$\begin{array}{c} L=\frac{1}{2}M+\frac{1}{2}N. \end{array}$$

Then, the weight parameter of the score can be expressed as follows:

(12) $$\begin{array}{c} W=1-\frac{L}{\sum_{i}^{h}L_{h}}. \end{array}$$

The percentile analysis method is a process of using judges to analyze qualitatively and then to score and evaluate each index according to the corresponding weight of the index. This method is simple to operate, but the subjective opinions of the judges of this method can interfere with the scoring results [17].

### 2.3. Fuzzy Analysis

Fuzzy is a commonly used analysis method, and statistical analysis of data using fuzzy allows causal analysis of conditions and targets fuzzy theory is developed on the basis of discrete mathematics, which is uncertain and extensive. Because fuzzy theory does not require precise analysis of the object under study, it is widely used. It is often used in sustainable environmental development, occupational health development of enterprise employees, and natural language processing. It can very well analyze the occupational health development and safety management issues of enterprise employees in a sustainable environment. The structure of fuzzy analysis is shown in Figure 3.

As can be seen from Figure 3, the general process of fuzzy analysis is as follows: determining the impact index, establishing the fuzzy matrix, analyzing the weight, obtaining the fuzzy judgment result, and optimizing the judgment result. Fuzzy theory is used in conjunction with AHP, using fuzzy analysis index factors to calculate the weight of judgment index through AHP [18].

### 2.4. Fuzzy AHP

Fuzzy AHP is to add fuzzy characteristics on the basis of AHP. The indicators that affect the occupational health development and safety management of enterprise employees are analyzed through fuzzy AHP. The structure model of fuzzy AHP is shown in Figure 4.

The analysis process of fuzzy AHP is as follows: determining the index, analyzing the index weight according to the judgment matrix, and analyzing the fuzzy decision-making [19].

There are *m* indicators *A*={*a*_1_, *a*_2_,…, *a*_*m*_}, the evaluation level of the indicators is *B*={*b*_1_, *b*_2_,…, *b*_*n*_}, and the weight set of each indicator is *W*={*w*_1_, *w*_2_,…, *w*_*m*_}.

(13) $$\begin{array}{c} \sum_{i=1}^{m}w_{i}=1. \end{array}$$

The membership degree of the impact index and the studied system is analyzed, so the membership degree of the index constitutes a fuzzy judgment matrix, and the fuzzy judgment matrix is expressed as follows:

(14) $$\begin{array}{c} H=\left[\begin{array}{cccc} h_{11} & h_{12} & \cdots & h_{1m}\\ h_{21} & h_{22} & \cdots & h_{2m}\\ \cdots & \cdots & \cdots \\ h_{n1} & h_{n2} & \cdots & h_{nm} \end{array}\right]. \end{array}$$

Burring the judgment level, let the decision-making level be C.

(15) $$\begin{array}{c} C=W\times H, \end{array}$$

(16) $$\begin{array}{c} C=\left(c_{1},c_{2},\ldots ,c_{n}\right). \end{array}$$

Here, *c*_*n*_ represents the weight of the *n*th index.

## 3. Experimental Design of Occupational Health and Safety Development of Enterprise Employees

### 3.1. Experimental Data

In order to analyze the relevant factors of occupational health development and safety management of enterprise employees from the perspective of sustainable environment, 500 enterprise employees in 50 enterprises were randomly investigated. And the causes of occupational diseases of enterprise employees were investigated without the employees' knowledge [20]. The causes of occupational diseases of enterprise employees are shown in Figure 5.

In Figure 5, the causes of occupational injuries of enterprise employees are mainly divided into four aspects: industrial wastewater, industrial waste, industrial waste gas, and industrial radiation. Through a questionnaire survey of environmental protection experts and occupational disease-attending physicians, the detailed reasons for occupational hazards of enterprise employees can be concluded [21]. The detailed occupational hazards of enterprise employees are shown in Table 2.

### 3.2. Experimental Design

The experiment will use the fuzzy analytic hierarchy process to analyze the indicators that affect the occupational health of enterprise employees in a sustainable environment [22, 23]. Then, a judgment matrix is constructed to analyze the impact weight of each index on the occupational health development and safety management of employees. Among them, the hazard type is represented by Y, and the hazard index is represented by X. The occupational health and safety development of enterprise employees with the largest weight among the four impact aspects is analyzed [24]. The judgment matrix of industrial wastewater and industrial waste impact indicators is shown in Table 3.

Performing an arithmetic mean solution on each column vector in Table 3, the relative weight of each index is obtained. The judgment matrix in Table 3 is tested for validity. The test result is as follows:

(17) $$\begin{array}{c} R=\frac{A}{B}=\frac{0.135}{1.41}=0.096. \end{array}$$

Because the obtained test result is less than 0.1, the judgment matrix of the impact indicators of industrial wastewater and industrial waste is effective. Similarly, the validity of the judgment matrix of industrial waste gas and industrial radiation and the weight of each index can be obtained. The weight results of all indicators are shown in Table 4.

In Table 4, the weights of the four types of criterion layers are 0.3, 0.25, 0.25, and 0.2, respectively. The indicators with the largest weights in each criterion layer are heavy metal wastewater, dust, hydrogen sulfide, and high-temperature radiation. Therefore, the experiment will analyze these four impact indicators for large enterprises and small enterprises, mainly by analyzing the change trend of the occupational safety of enterprise employees and the career development potential of enterprise employees when the gradient of the indicators changes [25].

## 4. Results and Discussion of the Impact of Indicators on the Occupation of Employees

### 4.1. Influence of Heavy Metal Wastewater

The discharge of heavy metal wastewater is the result of improper treatment of industrial wastewater by enterprises. Heavy metal wastewater contains substances that are harmful to human body. Long-term exposure to heavy metal wastewater environment is very harmful to people [26].  Figure 6 shows the effect of the content of heavy metal wastewater with different gradients on both large- and small-scale enterprise employees.

In Figure 6, when the concentration of heavy metal wastewater is less than 0.05 mg/L, the occupational safety and development of employees in mass-scale enterprises have a high level, and when the concentration of heavy metal wastewater is greater than 0.05 mg/L, the safety and development of this method are severely limited [27]. When the concentration of heavy metals is 0.10 mg/L, the occupational safety of employees in the two companies is 32% and 38%, respectively. The career development potential is 21% and 30%, respectively. Therefore, sustainable environmental strategies should be adhered to, so that the discharge of wastewater can effectively improve the occupational safety and development of employees.

### 4.2. Influence of Dust

Dust is a substance that is easily produced in industrial production and is harmful to human body. When the concentration of dust reaches a certain amount, it is very easy to cause employees to suffer from tuberculosis and other diseases. The concentration of dust with different gradients is set, and the effect of different concentrations of dust on both large- and small-scale enterprise employees is shown in Figure 7.

In Figure 7, when the dust concentration is below 4 mg/m^3^, the occupational safety and development of employees of the enterprise can reach a level of more than 70%, whether it is a large or a small enterprise. However, when the dust concentration is greater than 4 mg/m3, the occupational safety and development of the employees of the enterprise are seriously threatened. The occupational safety and development of employees in the two types of enterprises drop sharply, reaching the lowest when the dust concentration is 7 mg/m3. The average enterprise security for both sizes is only 36%, and the average career development force is 35%. Reducing the generation of dust in a sustainable environment can effectively improve the occupational health development and safety management of enterprise employees [28].

### 4.3. Influence of Hydrogen Sulfide Gas

In chemical enterprises, the generation of toxic gases is very common. Although there are professional protective measures, the harm of toxic gases to enterprise employees cannot be avoided. Among them, hydrogen sulfide is a common enterprise hazardous gas. Detecting the concentration of hydrogen sulfide gas in different enterprises, the influence of the concentration of hydrogen sulfide gas on both large- and small-scale enterprise employees is shown in Figure 8.

In Figure 8, the turning point of the change in employee occupational safety and development is when the concentration of hydrogen sulfide gas is 4.6 ppm. When the concentration of hydrogen sulfide gas is less than 4.6 ppm, the hydrogen sulfide gas does not cause harm to the human body or the harm caused is not high. The occupational safety of employees of both large- and small-scale enterprises can reach more than 70%, and the development power of employee enterprises can also reach more than 60%; however, when the concentration of hydrogen sulfide gas is greater than 4.6 ppm, the occupational safety and development ability of employees in both enterprises plummet, which has threatened the health of employees. The minimum average occupational safety is 16.5%, and the average enterprise development power is 30%. Reducing the generation of toxic gases such as hydrogen sulfide in the perspective of sustainable environment can effectively protect the occupation of enterprise employees.

### 4.4. Influence of High-Temperature Radiation

High-temperature radiation is a common problem in the industrial production of enterprises. The detection of high-temperature radiation duration is carried out on both large- and small-scale enterprises. The results of the impact of high-temperature radiation on the occupation of enterprise employees under different durations of high-temperature radiation are shown in Figure 9.

In Figure 9, when the employees of the enterprise are protected by professional protective clothing, the impact of high-temperature radiation on the employees of the enterprise for 2 consecutive hours is not very large. At this time, the average occupational safety of employees in both the enterprises is 68%, and the average employee career development ability is 72%. When the duration of high-temperature radiation exceeds 2 hours, it will pose a serious threat to the occupational safety of employees. When the duration of high-temperature radiation increases, the occupational safety and development of employees of the enterprise will plummet, and the lowest at 6 hours. At this time, the average occupational safety of enterprises of both sizes is 20.5%, and the average development force is 29%. Reducing the high-temperature radiation of enterprises under the sustainable environmental development strategy can improve the occupational health development and safety management of enterprise employees.

## 5. Conclusion

This paper analyzed the indicators that affect the occupational health development and safety management of employees in a sustainable environment through the fuzzy analytic hierarchy process. It summarized four aspects: industrial wastewater, industrial waste, industrial waste gas, and industrial radiation. Using the judgment matrix to analyze the index weight of this impact, four largest weight indexes are obtained. The impact index is set to gradient to analyze the occupational safety and development of the employees of the enterprise. The test results showed that when the concentration of the four indicators—heavy metal wastewater, dust, hydrogen sulfide gas, and high-temperature radiation—is low, the occupational safety and development of enterprise employees is higher; however, when the concentration of these indicators increases, the occupational safety and development ability of employees cannot be guaranteed. The average occupational safety of enterprise employees is 23%, and the average development ability is 25%. Adhering to sustainable environmental development and effectively reducing the generation of waste liquid, waste, waste gas, and radiation can not only effectively protect the environment but also guarantee the occupation of enterprise employees, so that the occupational health and safety of enterprise employees can develop. However, the analysis of the impact indicators in this paper is not detailed enough; for example, the types of dust can also be analyzed in detail to improve more accurate experimental data. Therefore, further details on the impact indicators will be the direction of future research.

## Figures and Tables

**Figure 1:** Structure diagram of occupational health development and safety management of enterprise employees.

**Figure 2:** AHP structure model diagram.

**Figure 3:** Fuzzy analysis structure diagram.

**Figure 4:** Structure model diagram of fuzzy AHP.

**Figure 5:** Causes of occupational diseases of employees in enterprises.

**Figure 6:** Impact of heavy metal wastewater: (a) occupational safety and (b) occupational development potential

**Figure 7:** Dust effect: (a) occupational safety and (b) occupational development potential

**Figure 8:** Influence of hydrogen sulfide gas: (a) occupational safety and (b) occupational development potential

**Figure 9:** Influence of high-temperature radiation: (a) occupational safety and (b) occupational development potential.

**Table 1:** Interpretation table of the meaning of judgment matrix.

Score	Influence relationship	Degree
1	Indicator 1 = Indicator 2	degree 0
2	Indicator 1 > Indicator 2	degree 1
3	Indicator 1 > Indicator 2	degree 2
4	Indicator 1 > Indicator 2	degree 3
5	Indicator 1 > Indicator 2	degree 4
6	Indicator 1 > Indicator 2	degree 5
7	Indicator 1 > Indicator 2	degree 6
8	Indicator 1 > Indicator 2	degree 7
9	Indicator 1 > Indicator 2	degree 8
Reciprocal	Indicator 1 < Indicator 2	Corresponding positive degree

**Table 2:** Detailed table of the occupation hazards of enterprise employees.

Hazardous objects	Hazard type	Hazard indicator
Occupational health development of enterprise employees	Industrial wastewater	Heavy metal wastewater
		Mercury wastewater
		Sulfuric acid wastewater
		Lead-containing wastewater
	Industrial waste	Dust
		Cinder
		Waste plastic
		Rubber waste
	Industry exhaust	Carbon monoxide
		Carbon dioxide
		Hydrogen sulfide
		Sulfur monoxide
	Industrial radiation	High-temperature radiation
		Infrared radiation
		Microwave radiation
		UV radiation

**Table 3:** Judgment matrix of impact indicators.

Y1 and Y2	X1	X2	X3	X4	X5	X6	X7	X8
X1	1	1/5	1/2	1	1/2	2	4	5
X2	5	1	2	5	3	4	1/2	3
X3	2	1/2	1	2	1/5	6	3	1/2
X4	1	1/5	1/2	1	1/3	1	1/4	4
X5	2	1/3	5	3	1	2	1/5	1/3
X6	1/2	1/4	1/6	1	1/2	1	4	2
X7	1/4	2	1/3	4	5	1/4	1	1/5
X8	1/5	1/3	2	1/4	3	1/2	5	1

**Table 4:** Weighting result table of each indicator.

Criterion layer	Indicator layer	Weights
Industrial wastewater	Heavy metal wastewater	0.12
	Mercury wastewater	0.04
	Sulfuric acid wastewater	0.08
	Lead-containing wastewater	0.06

Industrial waste	Dust	0.09
	Cinder	0.05
	Waste plastic	0.05
	Rubber waste	0.06

Industry exhaust	Carbon monoxide	0.06
	Carbon dioxide	0.05
	Hydrogen sulfide	0.08
	Sulfur monoxide	0.06

Industrial radiation	High-temperature radiation	0.06
	Infrared radiation	0.05
	Microwave radiation	0.05
	UV radiation	0.04

## Data Availability

No data were used to support this study.
